The article "Redox Imbalance in CD4+ T Cells of Relapsing-Remitting Multiple Sclerosis Patients" was published in 2020. Journal: Oxid Med Cell Longev.

# Redox Imbalance in CD4+ T Cells of Relapsing-Remitting Multiple Sclerosis Patients

**DOI:** 10.1155/2020/8860813

**Published:** 2020-12-02

**Authors:** Mohammad Javad Tavassolifar, Abdorreza Naser Moghadasi, Behnaz Esmaeili, Omid Sadatpour, Mohammad Vodjgani, Maryam Izad

**Affiliations:** ^1^Immunology Department, School of Medicine, Tehran University of Medical Sciences, Tehran, Iran; ^2^MS Research Center, Neuroscience Institute, Tehran University of Medical Sciences, Tehran, Iran; ^3^Immunology, Asthma and Allergy Research Institute (IAARI), Tehran University of Medical Sciences, Tehran, Iran

## Abstract

As a prevalent autoimmune disease of the central nervous system in young adults, multiple sclerosis (MS) is mediated by T cells, particularly CD4+ subsets. Given the evidence that the perturbation in reactive oxygen species (ROS) production has a pivotal role in the onset and progression of MS, its regulation through the antioxidant molecules is too important. Here, we investigated the level of the redox system components in lymphocytes and CD4+ T cells of MS patients. The study was performed on relapsing-remitting MS (RRMS) patients (*n* = 29) and age- and sex-matched healthy controls (*n* = 15). Peripheral blood mononuclear cells (PBMCs) were cultured and stimulated by anti-CD3/CD28. The level of ROS, anion superoxide (O_2_^−^), and L-𝛾-glutamyl-Lcysteinylglycine (GSH) was measured by flow cytometry in lymphocytes/CD4+ T cells. The gene expression level of gp91phox, catalase, superoxide dismutase 1/2 (SOD), and nuclear factor-E2-related factor (Nrf2) was also measured by real-time PCR. We found that lymphocytes/CD4+ T cells of RRMS patients at the relapse phase significantly produced higher levels of ROS and O_2_^−^ compared to patients at the remission phase (*P* value < 0.001) and healthy controls (*P* value < 0.001 and *P* value < 0.05, respectively). Interestingly, the gene expression level of gp91phox, known as the catalytic subunit of the NADPH oxidase, significantly increased in MS patients at the relapse phase (*P* value < 0.05). Furthermore, the catalase expression augmented in patients at the acute phase (*P* value < 0.05), while an increased expression of SOD1 and Nrf2 was found in RRMS patients at relapse and remission phases (*P* value < 0.05). The increased production of ROS in CD4+ T cells of RRMS patients highlights the importance of amplifying antioxidant components as an efficient approach to ameliorate disease activity in MS patients.

## 1. Introduction

Multiple sclerosis (MS) is an inflammatory and immune-mediated disease of the central nervous system (CNS) common in young adults [1]. Whereas MS prevalence has an increasing trend in the world, disease prevention and management could reduce its socioeconomic impact [2]. Genetic factors, together with environmental stimuli, play a substantial role in MS susceptibility [1]. To date, numerous studies pointed to the central role of CD4+ T cell populations in the disease pathogenesis. Following the recognition of myelin-like peptides, circulating CD4+ T cells infiltrate into the CNS, leading to demyelination through various effector molecules [3, 4]. Besides, a growing body of evidence speculated the involvement of oxidative stress in the initiation and progression of many autoimmune diseases, including MS [5, 6].

The article "Redox Imbalance in CD4+ T Cells of Relapsing-Remitting Multiple Sclerosis Patients" was published in 2020. Journal: Oxid Med Cell Longev.

The term “oxidative stress” is described as a disturbed balance between reactive oxygen species (ROS) and antioxidant molecules [7]. ROS is referred to as a group of molecules produced through reduction-oxidation (redox) reactions or electronic excitation. Superoxide anion (O_2_^·-^), hydroxyl radical (^·^OH), and hydrogen peroxide (H_2_O_2_) are major ROS, which are prominently produced by nicotinamide adenine dinucleotide phosphate oxidase (NADPH oxidases, NOX) [8, 9]. ROS is involved in several biological activities as second messengers in the signaling cascade, particularly in the immune system and CNS [8]. Previous studies demonstrated that ROS comprehensively influences T cell differentiation and proliferation [10, 11]. Under normal metabolism, the antioxidant system controls ROS-mediated signaling pathways [7]. The accumulation of ROS in NOX-deficient or early response gene X-1 (IEX-1) knockout mice enhanced Th17 [12, 13]. Besides, the decreased expression of CD25, CD69, and production of IL-2 has been found in CD4+ T cells treated with transcription factor nuclear factor-E2-related factor (Nrf2) activators [14].

The antioxidant system employed enzymatic and nonenzymatic antioxidant scavenging elements. While the former mainly include superoxide dismutase (SOD), catalase (CAT), glutathione peroxidase (GPx), glutathione reductase (GR), and thioredoxin reductase, which are regulated by Nrf2. The latter includes reduced L-𝛾-glutamyl-Lcysteinylglycine (GSH) [15, 16].

To date, the significance of oxidative stress in the pathophysiology of autoimmune diseases, particularly MS, is well explained. Data from blood samples of RRMS patients suggested increased ROS production and impaired antioxidant capacity, which were accompanied by nuclear factor kappa beta (NF-*κβ*) stimulation [17]. The higher level of superoxide is also associated with microglia-induced myelin degradation [18]. The involvement of NOX in experimental autoimmune encephalopathy (EAE), the animal model of MS, has also been reported [19]. Noteworthily, using a microarray, an upregulated expression of both NOX and Nrf2 was reported in activated MS lesions [20, 21]. Also, a significant reduction of SOD and GPX activities has been shown in CD4+ T cells isolated from RRMS patients [22]. Dimethyl fumarate (DMF) exerts its effect on MS progression through the activation of the Nrf2 pathway [23, 24].

The article "Redox Imbalance in CD4+ T Cells of Relapsing-Remitting Multiple Sclerosis Patients" was published in 2020. Journal: Oxid Med Cell Longev.

Regarding the importance of both oxidative stress and CD4+ T cells in MS pathogenesis, we decided to investigate the oxidant and antioxidant capacity of lymphocytes/CD4+ T cells in RRMS patients, at relapse and remission phases, in comparison to healthy controls.

## 2. Materials and Methods

### 2.1. Participants

Twenty-nine RRMS patients, diagnosed based on McDonald's diagnostic criteria for MS [25] considering patients' history and magnetic resonance imaging (MRI), participated in the present study. Fourteen patients were at the relapse phase (female = 11 and male = 3, mean age = 35.14 ± 2.6) and fifteen patients at the remission phase (female = 12 and male = 3, mean age = 31.6 ± 1.8). All patients were referred to the Iranian Center of Neurological Research in Sina General Hospital, Tehran University of Medical Sciences, Tehran, Iran. The inclusion criteria for patients in the acute phase include not receiving any disease-modifying therapies (DMTs) and corticosteroid for at least three prior months. All of the patients in the remission phase have received IFN-*β*. Moreover, fifteen healthy controls (12 females and 3males, mean age = 30.5 ± 1.2) enrolled in the study were defined as individuals who had no history of MS or other autoimmune and inflammatory diseases.

Both patients and healthy controls have not received any antioxidant supplements for at least four weeks before sampling. The participants were informed about the procedure of the study, and informed consent was obtained from them. All participants were of Iranian origin. The study was approved by the ethics committee of Tehran University of Medical Sciences (TUMS), “IR.TUMS.MEDICINE.REC.1398.044.”

### 2.2. Cell Culture

Peripheral blood mononuclear cells (PBMCs) were isolated by Ficoll density gradient sedimentation (Lymphodex, Inno-Train, Germany). The PBMCs were cultured at a concentration of 1 × 10^6^ cells/well and activated with soluble anti-human CD3/CD28 mAb (0.1 *μ*g/mL) (Mabtech, Sweden) for 72 hours in RPMI 1640 medium (Gibco, USA), containing 10% (*V*/*V*) FBS (Biosera-France, FB-1001) and 1% Penicillin-Streptomycin Solution 100x (Biosera-France) and incubated at 37°C in a humidified 5% CO_2_.

### 2.3. Flow Cytometry

To evaluate the intracellular ROS production level, ROS and superoxide detection assay kit (ab139476, USA) was used. According to the instruction manual, approximately 25 × 10^4^ cultured cells were harvested, washed, and incubated with permeable green probe (reacts with hydrogen peroxide, peroxynitrite (ONOO⎯), hydroxyl radicals (HO), nitric oxide (NO), and peroxyradical (ROO)) and orange probe (reacts especially with superoxide (O_2_^⎯^)) for 30 minutes at 37°C. Also, the GSH level as an antioxidant molecule was measured using a GSH assay kit (ab112132, USA). Briefly, after cell culture, 5 × 10^5^ cells were harvested, washed, and incubated with thiol green dye for 20 minutes at 24°C. To analyze intracellular ROS/superoxide and GSH in CD4+ T cells, anti-human CD4-APC (Biolegend, USA) was added to the cells previously stained with ROS/superoxide and GSH probes and assessed by flow cytometry. ROS/superoxide and GSH production was calculated based on the difference between the mean fluorescence intensity of stimulated and unstimulated cells.

The article "Redox Imbalance in CD4+ T Cells of Relapsing-Remitting Multiple Sclerosis Patients" was published in 2020. Journal: Oxid Med Cell Longev.

### 2.4. Real-Time PCR

To assess gene expression levels of gp91phox, NADPH oxidase subunit, and antioxidant enzymes, including CAT, SOD1, SOD2, and Nrf2, total RNA was extracted from stimulated cells by RNX-plus solution (RN7713C, Sinaclon, Iran) according to the manufacturer's instruction. RNA concentration and integrity were measured using NanoDrop (Thermo Fisher). The isolated RNA was treated with DNase I (Fermentas, USA) to eliminate genomic DNA. Subsequently, cDNA was synthesized using a cDNA synthesis kit (Thermo Fisher Scientific, USA). Real-time PCR was performed on an ABI step one plus real-time PCR system (Applied Biosystem) using 2x SYBR Green qPCR Mix plus (ROX) (Ampliqone, Denmark). Relative expression levels of these genes were normalized by 18s rRNA as a housekeeping gene and calculated by the 2−*ΔΔ*Ct method. The sequences of primers are listed in Table 1.

### 2.5. Statistical Analysis

All analysis was performed by Statistical Package for the Social Sciences (SPSS) software version 21.0 (SPSS Inc.; Chicago, IL, US). One-way ANOVA and Tukey's post hoc test were used for comparing superoxide and GSH levels in CD4+ T cells between RRMS patients and healthy controls. Moreover, the analysis of gene expression between the studied groups was performed using the REST software (version 2009). Data are expressed as the mean ± SD. Results with *P* value less than 0.05 were considered significant.

## 3. Results

For evaluation of the ROS and antioxidant levels in lymphocytes/CD4+ T cells of MS patients, 29 RRMS patients at relapse and remission phases and 15 healthy controls were examined in the current study (Table 2).

### 3.1. ROS/Superoxide and GSH Production Increased in CD4+ T Cells of RRMS Patients

For investigating oxidative stress phenomena in RRMS patients, we analyzed ROS/superoxide production and GSH intracellular level in unstimulated and stimulated lymphocytes and CD4+ T cells. Lymphocytes were first gated on a forward vs. side scatter dot plot. CD4+ T cells producing ROS/superoxide and GSH were analyzed on gated lymphocytes. The gating strategy to determine ROS/superoxide and GSH production in gated lymphocytes and CD4+ T cells is shown in Figures 1 and 2.

The article "Redox Imbalance in CD4+ T Cells of Relapsing-Remitting Multiple Sclerosis Patients" was published in 2020. Journal: Oxid Med Cell Longev.

Significant higher production of ROS was observed in lymphocytes and CD4+ T cells in RRMS patients at the relapse phase compared to patients at the remission phase and healthy individuals (*P* value < 0.02 and *P* value < 0.001, respectively) (Figures 3(a) and 3(b)). The level of ROS was also increased in RRMS patients at the remission phase compared to healthy individuals (*P* value < 0.05). Furthermore, we observed an elevated O_2_^−^ production in lymphocytes of RRMS patients at the relapse phase in comparison to the remission phase (*P* value < 0.05) (Figure 3(c)), while O_2_^−^ showed increased production in CD4+ T cells of RRMS patients at the relapse phase compared to patients at the remission phase and healthy individuals (*P* value = 0.002 and *P* value < 0.001, respectively) (Figure 3(d)).

We also identified a significantly higher level of GSH in lymphocytes of RRMS patients at relapse and remission phases than healthy individuals (*P* value < 0.05 and *P* value < 0.001, respectively). Interestingly, the GSH level increased in lymphocytes of RRMS patients at the remission phase when compared with the relapse phase (*P* value = 0.004) (Figure 3(e)). Moreover, intracellular GSH levels are augmented in CD4+ T cells of RRMS patients at relapse and remission phases than healthy individuals (*P* value > 0.05 and *P* value < 0.001, respectively) (Figure 3(f)).

### 3.2. Gene Expression of Antioxidant Molecules Increased in RRMS Patients

To have better insights regarding the role of oxidative stress molecules in MS, we also examined the balance between oxidants (NOX-gp91phox) and antioxidants (CAT, SOD1, SOD2, and Nrf2) at the gene expression level in activated lymphocytes. There was a significant increase in gp91phox gene expression in patients at the relapse phase compared to healthy subjects (*P* value < 0.05). The expression level of CAT was increased in RRMS patients at the relapse phase in comparison to patients at the remission phase and healthy subjects (*P* value < 0.05). The SOD1 upregulated in RRMS patients at relapse and remission phases in comparison to healthy controls (*P* value = 0.003 and *P* value < 0.05, respectively). Although the SOD2 gene expression increased at the relapse phase than healthy individuals, it was not significant (*P* value = 0.08). Furthermore, we identified a higher expression of Nrf2 in RRMS patients at relapse and remission phases than healthy controls (*P* value < 0.05) (Figure 4).

The article "Redox Imbalance in CD4+ T Cells of Relapsing-Remitting Multiple Sclerosis Patients" was published in 2020. Journal: Oxid Med Cell Longev.

## 4. Discussion

As a common inflammatory disease of the CNS, MS is mainly mediated by pathogenic T cells, particularly CD4+ T cells [3]. It is well known that oxidative stress has a critical role in the development of inflammatory responses in autoimmune diseases such as MS [8]. However, little is known about the balance of oxidant and antioxidant molecules in CD4+ T cells of RRMS patients at different stages of the disease. In the current study, for the first time, we identified the occurrence of the oxidative burst in CD4+ T cells of RRMS patients at the relapse phase.

Several studies have pointed to the alteration of ROS and O_2_^·-^, or other oxidative stress-related markers in several autoimmune diseases [13, 26]. Our recent research has also shown the increased production of ROS in memory CD4+ T cells of psoriasis patients [27]. Here, we demonstrated that ROS and O_2_^·-^ were produced at a higher level in CD4+ T cells of RRMS patients at the relapse phase compared to the remission phase and healthy controls. The increased ROS production and impaired antioxidant capacity were also identified in blood samples of RRMS patients, which ultimately lead to activation of NF-*κβ* [17]. Through inducing the expression of cell adhesion molecules (e.g., ICAM-1, VCAM-1, and PECAM-1) at endothelial cells of BBB, it is suspected that ROS might increase the migration of inflammatory lymphocytes, particularly T cells, to the CNS [28]. Interestingly, microglia-induced myelin degradation is also linked to the abundant amounts of oxidant molecules like superoxide [18]. ROS is also implicated in the activation and differentiation of T cells, key orchestrators in MS pathogenesis [29]. In IEX-1 knockout mice, ROS-mediated signaling has been shown to increase IL-17 production following T cell activation [13].

In addition to the mitochondrial respiratory chain, the production of ROS from molecular oxygen is mediated by a family of enzymes called NADPH oxidases (NOXes) [8]. Among different isoforms, NOX2 has been proposed as a key component in MS and EAE pathogenesis. Of note, the upregulated expression of gp91phox, the catalytic subunit of NOX2, has been found in activated microglia and macrophages in early MS lesions [20]. The increased expression of gp91phox was also demonstrated in MOG-induced EAE [19]. Consistent with previous studies, we observed a significant rise in gp91phox expression in CD4+ T cells of RRMS patients at the active phase. Perhaps, NOX2-derived ROS in CD4+ T cells contributes to the MS pathogenesis.

The article "Redox Imbalance in CD4+ T Cells of Relapsing-Remitting Multiple Sclerosis Patients" was published in 2020. Journal: Oxid Med Cell Longev.

Since the activation of oxidant molecules is proposed as one of the major causes of inflammation in MS pathogenesis, endogenous antioxidant enzymes may play a pivotal role to control tissue damage in the disease. Catalase and SOD1/SOD2 as the major enzymatic antioxidants in ROS detoxification have gained particular attention [30]. We detected higher expression of the CAT gene in RRMS patients at the active phase compared to the remission phase as well as healthy controls. Emamgholipour et al. also demonstrated a significant increase in mRNA expression and activity of catalase in the PBMCs of RRMS patients in comparison to controls [31]. Previously, the increased mRNA expression and activity of peroxisomal enzyme catalase have been reported in grey and white matter of MS patients, predominantly in microglial cells [32, 33]. Some studies also reported increased catalase activity in CSF and plasma of MS patients [34, 35]. In the context of SOD, our results identified overexpression of SOD1 in CD4+ T cells of RRMS patients, but the SOD2 expression level was similar among studied groups. According to the previous research, intracellular SOD1 protein as well as mRNA in PBMCs is increased by IFN-*β* 1b therapy [36]. The upregulated expression of SOD1 is reported in blood and lesions of acute and chronic MS patients [37, 38]. However, a study showed a significant reduction of SOD and stable activity of CAT in CD4+ T cells isolated from RRMS patients [22]. Other studies showed no significant platelet SOD1 and SOD2 activity differences between MS patients and healthy controls [39].

In addition to enzymatic antioxidants, the antioxidant system comprises small molecules. A reduced form of glutathione, GSH, one of the electron donors, mediates defense against ROS [30]. Here, the augmented production of GSH in CD4+ T cells was revealed in RRMS patients, both at the relapse and remission phases. Concordant with this, the increment of GSH levels in the blood of MS patients was reported [17]. Inconsistently, several studies reported a lower level or no statistically significant differences of CSF or whole blood GSH level in MS patients [35, 40].

To maintain the redox balance in the cells, the antioxidant system should be regulated. In this regard, the importance of NF-E2-related factor 2 (Nrf2) as a key regulator of the antioxidant system is well described [41]. Earlier data also suggested that Nrf2 deficiency or lower expression level could exacerbate the disease pathology in EAE [42, 43]. In our study, we observed a higher expression of Nrf2 in CD4+ T cells of RRMS patients compared to healthy individuals. Recently, high Nrf2 expression in active lesions of acute, relapsing, and progressive MS lesions, predominantly in oligodendrocytes, has been reported [21]. The upregulated expression of Nrf2 in the nucleus and the cytoplasm of infiltrating macrophages and astrocytes of active MS lesions has been demonstrated [44]. Remarkably, Gopal et al. provide the first evidence regarding the activation of Nrf2 pathways in DMF-treated MS patients [24]. Subsequently, inducing an anti-inflammatory shift in circulating immune cell subsets following the upregulation of Nrf2 expression was shown in MS patients treated with DMF [45].

The article "Redox Imbalance in CD4+ T Cells of Relapsing-Remitting Multiple Sclerosis Patients" was published in 2020. Journal: Oxid Med Cell Longev.

## 5. Conclusion

In the present study, for the first time, we highlighted the perturbation of the redox system homeostasis in lymphocytes and CD4+ T cells of RRMS patients. In parallel with the augmented production of ROS and superoxide anion, NOX-gp91phox expression was also increased in RRMS patients. Besides, we observed a higher expression level of antioxidant components such as catalase, GSH, and SOD1 and Nrf2. It seems that antioxidant molecules are activated to regulate the redox system in T cells of MS patients. However, the activation is not sufficient to overcome ROS. So, the oxidative burst might ultimately lead to the polarization of inflammatory T cells. Therefore, our findings suggest reducing CD4+ T lymphocyte dysfunctions by increasing antioxidant activity, and their response to oxidative stress may be effective for ameliorating MS symptoms.

## Figures and Tables

**Figure 1:** Representative gating strategy for ROS/superoxide and GSH production in lymphocytes of RRMS patients and healthy controls. ROS/superoxide and GSH production among (a) unstimulated and (b) stimulated lymphocytes was determined by flow cytometry in unstained (green line), healthy controls (orange line), and RRMS patients at relapse and remission phases (red and blue lines, respectively).

**Figure 2:** Representative gating strategy for ROS/superoxide and GSH production in CD4+ T cells of RRMS patients compared to healthy controls. ROS/superoxide and GSH production among (a) unstimulated and (b) stimulated CD4+ T cells was determined by flow cytometry in unstained (green line), healthy controls (orange line), and RRMS patients at relapse and remission phases (red and blue lines, respectively).

**Figure 3:** ROS/superoxide production and GSH intracellular level measured by flow cytometry in lymphocytes and CD4+ T cells of RRMS patients and healthy controls. ROS/superoxide production and GSH intracellular levels in (a) lymphocytes and (b) CD4+ T cells isolated from RRMS patients at relapse and remission phases and healthy controls. One-way ANOVA was used to examine the difference across studied groups. Tukey's post hoc test was used to compare means. ^∗^*P* value ≤ 0.05; ^∗∗∗^*P* value ≤ 0.001. MFI: mean fluorescence intensity.

The article "Redox Imbalance in CD4+ T Cells of Relapsing-Remitting Multiple Sclerosis Patients" was published in 2020. Journal: Oxid Med Cell Longev.

**Figure 4:** The oxidant and antioxidant molecules examined by real-time PCR in activated lymphocytes of RRMS patients and healthy controls. The gene expression level of (a) gp91phox, (b) CAT, (c) SOD1, (d) SOD2, and (e) Nrf2 was investigated in RRMS patients at relapse and remission phases and healthy controls. One-way ANOVA was used to examine the difference across studied groups. To compare means, Tukey's post hoc test was used. ^∗^*P* value ≤ 0.05; ^∗∗∗^*P* value ≤ 0.001.

**Table 1:** Primers used for gene expression analysis through real-time PCR.

Gene name	Forward primer (5′ → 3′)	Reverse primer (5′ → 3′)
gp91phox	CTGGAAACCCTCCTATGACTTG	GTGATGACCACCTTCTGTTGAG
CAT	TGCTGAATGAGGAACAGAGGAA	CCTCACAGATTTGCCTTCTCC
Nrf2	CCATTCCTGAGTTACAGTGTCT	CTGTGGAGAGGATGCTGC
SOD1	AGCGAGTTATGGCGACGAAG	CAGCCTGCTGTATTATCTCCA
SOD2	CTCAGGTTGGGGTTGGCT	TGAAGGTAGTAAGCGTGCTCC
18s rRNA	GTAACCCGTTGAACCCCATT	CCATCCAATCGGTAGTAGCG

**Table 2:** Characteristic of MS patients and healthy controls and some inclusion and exclusion criteria.

Characteristics	RRMS patients		Controls (*n* = 15)
	Relapse phase (*n* = 14)	Remission phase (*n* = 15)	
Inclusion criteria	Relapsed RRMS patients	Patients received IFN-*β*	Healthy adults
Exclusion criteria	History of immunosuppressive drugs in the previous 3 months	History of other drugs	History of autoimmune diseases
Sex (female/male)	11/3	12/3	12/3
Age (years)	35.14 ± 2.6	31.6 ± 1.8	30.5 ± 1.2
EDSS score	2.3 ± 0.5	2.35 ± 0.7	—
Disease duration (years)	2.5 ± 0.9	4.5 ± 1.1	—

## Data Availability

No data were used to support this study.
